The article "miR-30a-5p Regulates Viability, Migration, and Invasion of Lung Adenocarcinoma Cells via Targeting ECT2" was retracted in 2023. Reasons: signs of a paper mill; suspected computer-generated content; unreliable results or conclusions; concerns about the data.

# miR-30a-5p Regulates Viability, Migration, and Invasion of Lung Adenocarcinoma Cells via Targeting ECT2

**DOI:** 10.1155/2021/6241469

**Published:** 2021-07-07

**Authors:** Sangsang Chen, Xuqing Zhu, Jing Zheng, Tingting Xu, Yinmin Xu, Feng Chen

**Affiliations:** ^1^Department of Pharmacy, The Children's Hospital, Zhejiang University School of Medicine, National Clinical Research Center for Child Health, Hangzhou 310000, China; ^2^Department of Gastroenterology, Taizhou Municipal Hospital, Taizhou 318000, China; ^3^Department of Respiratory Medicine, Taizhou Municipal Hospital, Taizhou 318000, China; ^4^Department of Respiratory Medicine, Affiliated Hospital of Shaoxing University, Shaoxing 312000, China

## Abstract

**Objective:**

The abnormal expression of epithelial cell transforming sequence 2 (ECT2) is often considered the driving factor for the growth and invasion of tumors. This study was performed to investigate the regulatory effect of miR-30a-5p and ECT2 on lung adenocarcinoma (LUAD), which provides a basis for the effective clinical treatment of LUAD.

**Methods:**

The mature miRNAs, expression data of mRNAs, and clinical data of LUAD were downloaded from The Cancer Genome Atlas (TCGA). The expression levels of ECT2 mRNA and miR-30a-5p in cancer cell lines were detected by qRT-PCR. Western blot was performed to test the expression of ECT2 protein. The targeting relationship between miR-30a-5p and ECT2 was verified by dual-luciferase assay. The CCK-8 method and Transwell assay were conducted to test the viability, migratory, and invasive abilities of cells.

**Results:**

ECT2 expression was upregulated in LUAD and was significantly correlated with the LUAD clinical stage and pathologic T stage, and the expression of its upstream regulatory gene miR-30a-5p was downregulated. miR-30a-5p targeted ECT2 in LUAD. Downregulation of ECT2 could inhibit the viability, migration, and invasion of LUAD cells, which could be reversed by simultaneously suppressing the expression of miR-30a-5p.

**Conclusion:**

Our results suggested that miR-30a-5p repressed the malignant progression of LUAD via downregulating ECT2. miR-30a-5p and ECT2 may be effective targets for LUAD patients.

## 1. Introduction

Lung cancer is a leading cause of cancer-related deaths worldwide, and lung adenocarcinoma (LUAD) takes up about 50% of all lung cancer cases, with an increasing trend year by year [1]. LUAD is a type of non-small-cell lung cancer (NSCLC), most of which originate from the bronchial mucosal epithelium, and a few originate from the large bronchial mucous glands. Generally, the disease progresses slowly and the initial symptoms are not obvious [2]. Despite the recent advances in diagnosis and treatment strategies of LUAD, treatment failures are still common in patients with advanced LUAD [3]. To solve this problem, many researchers have carried out in-depth research and investigation. Early studies on genetics and epigenetics of LUAD reveal that epithelial cell transforming sequence 2 (ECT2) is differentially expressed in both adenocarcinoma *in situ* (AIS) and early invasive adenocarcinoma [4], suggesting that ECT2 may be a new entry point for LUAD treatment.

The article "miR-30a-5p Regulates Viability, Migration, and Invasion of Lung Adenocarcinoma Cells via Targeting ECT2" was retracted in 2023. Reasons: signs of a paper mill; suspected computer-generated content; unreliable results or conclusions; concerns about the data.

ECT2 is the guanine nucleotide exchange factor (GEF) of GTPase protein of the Rho family. ECT2 protein includes a C-terminal GEF domain that catalyzes the GEF activity, an N-terminal domain that regulates the GEF activity and localization, and a central S domain with two nuclear localization signals required for ECT2 nuclear localization [5]. In normal cells, ECT2 is located in the nucleus during interphase and distributed into the cytoplasm after the nuclear membrane rupture in prometaphase, then, cell division is stimulated by activating GTPase RhoA [6]. Studies demonstrate that ECT2 plays a promoting role in the malignant progression of cancers such as breast cancer [7], gastric cancer [8], and pancreatic cancer [9]. In lung cancer, many studies found that ECT2 is associated with lung cancer progression. For example, Shi et al. [10] found by genome-scale analysis that ECT2 has diagnostic and prognostic value in lung cancer. Bai et al. [11] collected data from clinical patients and found that ECT2 is markedly highly expressed in NSCLC and is correlated with the clinicopathological characteristics and prognosis of the patients.

Although there have been a large number of studies on the promoting effect of high expression of ECT2 on the malignant progression of LUAD, the specific pathogenic mechanism of ECT2 on LUAD remains unclear. In this study, we started by analyzing ECT2 and found its upstream regulatory gene miR-30a-5p through bioinformatics analysis. The function of ECT2 and miR-30a-5p in LUAD cells and the potential regulatory relationship between the two were studied through *in vitro* experiments. Finally, we manifested that miR-30a-5p can regulate the expression of ECT2 to inhibit LUAD progression, which provides a new therapeutic target for the treatment of LUAD.

## 2. Materials and Methods

### 2.1. Bioinformatics Analysis

The mature miRNAs of LUAD (normal: 46, tumor: 521), expression data of mRNA (normal: 59, tumor: 535), and clinical data were downloaded from TCGA (https://portal.gdc.cancer.gov/). The differential analysis of miRNAs and mRNAs in the normal group and tumor group was carried out by the edgeR package (∣logFC | >1.5, *p*_adj_ < 0.05) to obtain the differentially expressed miRNAs and mRNAs. The target mRNA was confirmed through the literature, and the relationship between the target mRNA and the clinical stage of LUAD was further analyzed by the data from TCGA-LUAD dataset. starBase (http://starbase.sysu.edu.cn/) was used to predict the upstream regulatory genes of the target mRNA, and the differentially expressed miRNAs with targeted binding sites on the target mRNA were obtained. Finally, correlation analysis was performed to determine the final upstream regulatory miRNA.

The article "miR-30a-5p Regulates Viability, Migration, and Invasion of Lung Adenocarcinoma Cells via Targeting ECT2" was retracted in 2023. Reasons: signs of a paper mill; suspected computer-generated content; unreliable results or conclusions; concerns about the data.

### 2.2. Cell Culture

The human bronchial epithelial cell line BEAS-2B (3153C0001000000175) and human LUAD cell lines Calu-3 (3111C0001CCC000032), SPC-A1 (3111C0001CCC000387), and NCI-H2009 (3111C0001CCC000383) were all purchased from the National Infrastructure of Cell Line Resource (NICR, China). All the cell lines were cultured in Dulbecco's modified Eagle's medium (DMEM) (Gibco, USA) containing 10% fetal bovine serum (FBS) (Gibco, USA) and were incubated in a constant temperature incubator at 37°C and 5% CO_2_ for future use.

### 2.3. Cell Transfection

The miR-30a-5p inhibitor (miR-inhibitor), NC-inhibitor, miR-30a-5p mimic (miR-mimic), NC-mimic, si-ECT2, and si-NC purchased from GenePharma (Shanghai, China) were transfected into the experimental cell lines using Lipofectamine 2000 (Invitrogen, Carlsbad, CA) according to the manufacturer's instructions. Cells were cultured in a complete medium at 5% CO_2_ and 37°C for future use. All cells should be cultured in the medium for at least 24 h before transfection. Cell transfection efficiency was detected by qRT-PCR after cells were transfected for 36 h.

### 2.4. RNA Extraction and qRT-PCR

Total RNA in cells was extracted by the TRIzol reagent (Invitrogen, Carlsbad, CA, USA). According to the manufacturer's instructions, miRNA was reversely transcribed into cDNA by the miRcute miRNA First-Strand cDNA Synthesis Kit (Tiangen, China) to detect miRNA expression. Similarly, in order to detect the expression of mRNA, the SuperScript III First-Strand Synthesis System Kit (Invitrogen, Carlsbad, CA) was used to reversely transcribe mRNA into cDNA. Finally, the SYBR® Green Real-Time PCR Master Mix (Takara Bio Inc., Shiga, Japan) was used to test the expression of miRNA and mRNA by qRT-PCR. U6 and *β*-actin were used as the internal reference for miRNA and mRNA, respectively. The calculation of relative expression levels was based on the 2^−*ΔΔ*Ct^ method, and the experiment was repeated three times. The primer sequences used in the experiment are demonstrated in Table 1.

### 2.5. CCK-8 Assay

The CCK-8 method was used to detect the cell viability in this study. The transfected cells were inoculated to 96-well plates at a density of 5 × 10^3^ cells per well; then, 10% CCK-8 (Beyotime Biotechnology, Shanghai, China) was added to the wells. The absorbance of the cells at 450 nm was measured with a spectrophotometer at 0 h, 24 h, 48 h, 72 h, and 96 h, respectively.

The article "miR-30a-5p Regulates Viability, Migration, and Invasion of Lung Adenocarcinoma Cells via Targeting ECT2" was retracted in 2023. Reasons: signs of a paper mill; suspected computer-generated content; unreliable results or conclusions; concerns about the data.

### 2.6. Transwell Assay

In cell migration assay, cells were resuspended in a serum-free medium. The cells were added to the Transwell upper chamber with 5 × 10^5^ cells/ml, and a complete medium containing 10% FBS was added to the lower chamber. After incubation at 37°C for 24 h, the unmigrated cells in the upper chamber were removed and crystal violet staining was performed, and excess crystal violet was discarded. After drying, the bottom membrane of the chamber was placed under a microscope for observation and counting. Transwell invasion assay was performed using an upper chamber coated with the Matrigel matrix, and the remaining procedures were the same as the cell migration assay.

### 2.7. Dual-Luciferase Reporter Assay

The synthesized ECT2 3′-UTR-wild type (WT) and ECT2 3′-UTR-mutant (MUT) were cloned into luciferase vectors to make the plasmid configuration complete. Cells were cultured in 48-well plates, and the ECT2 3′-UTR-WT or ECT2 3′-UTR-MUT plasmid vectors were cotransfected with the miR-mimic or NC-mimic using the Lipofectamine 3000 reagent (Invitrogen, Carlsbad, CA) into the cells. The Renilla luciferase expression vector pRL-TK (Takara, Dalian, China) was used as the internal reference. Luciferase assay reagents (Promega, Fitchburg, WI, USA) were used to detect luciferase activity at 48 h after transfection.

### 2.8. Western Blot Assay

The radioimmunoprecipitation assay (RIPA) buffer with 0.1% phenylmethylsulfonyl fluoride (PMSF) was used, and the cells were placed on ice for lysis for 20 min. After centrifugation (12,000 g, 4°C, and 10 min), the supernatant was transferred to a new EP tube to obtain the total protein products of cells. The protein concentration of the samples was determined by the BCA method, and protein was conducted according to different protein concentrations. The proteins were separated by sodium dodecyl sulfate-polyacrylamide gel electrophoresis (SDS-PAGE) and were immediately transferred to a polyvinylidene difluoride (PVDF) membrane treated with methanol. Under the condition of 4°C, the membrane was added with 5% skim milk powder and incubated overnight. Subsequently, the primary anti-ECT2 antibody (Abcam, UK) and anti-glyceraldehyde 3-phosphate dehydrogenase (GAPDH) antibody (Abcam, UK) were added to the membrane and incubated at room temperature for 2 h. Then, the membrane was incubated for 30 min at the same condition of room temperature with the secondary antibody goat anti-rabbit IgG (Abcam, UK). GAPDH was used as the internal reference. An optical luminometer (GE, USA) was used for scanning and development; then, photos were taken.

The article "miR-30a-5p Regulates Viability, Migration, and Invasion of Lung Adenocarcinoma Cells via Targeting ECT2" was retracted in 2023. Reasons: signs of a paper mill; suspected computer-generated content; unreliable results or conclusions; concerns about the data.

### 2.9. Data Statistics

All data were processed by Prism 8.0 statistical software. Measurement data were expressed in the form of mean ± standard deviation. The comparison between two groups was detected by *t*-test, and the comparison between multiple groups was assessed by one-way analysis of variance (ANOVA). *p* < 0.05 indicated that the difference was statistically significant.

## 3. Results

### 3.1. ECT2 Is Upregulated in LUAD and Is Related to LUAD Staging

In order to explore the expression of ECT2 in LUAD, bioinformatics analysis was first performed to obtain 3611 differentially expressed mRNAs (Figure 1(a)), and ECT2 was highly expressed in LUAD tissue (Figure 1(b)). The survival analysis manifested that the survival time of patients with high expression of ECT2 was notably shorter than that of patients with low expression of ECT2 (Figure 1(c)). Subsequently, through further analysis of the data in TCGA-LUAD dataset, we found that ECT2 was markedly correlated with the LUAD clinical stage and pathologic T stage (Figures 1(d) and 1(e)). Then, qRT-PCR was performed to detect ECT2 expression in the human bronchial epithelial cell line BEAS-2B and LUAD cell lines (Calu-3, NCI-H2009, and SPC-A1). The results showed that compared to human bronchial epithelial cells, ECT2 was upregulated in LUAD cells (Figure 1(f)). Among LUAD cells, ECT2 presented the biggest expression difference in the cell line NCI-H2009; thus, we chose the cell line NCI-H2009 for further experiments.

### 3.2. Downregulating ECT2 Inhibits the Viability, Migration, and Invasion of LUAD Cells

In order to investigate the effect of ECT2 expression on LUAD, we first conducted qRT-PCR and Western blot assay to detect mRNA expression and protein expression of ECT2 in NCI-H2009 cells after transfection with si-ECT2, and the results manifested that the expression levels of mRNA and protein of ECT2 both decreased (Figures 2(a) and 2(b)). Subsequently, CCK-8 and Transwell migration and invasion assays were performed to test the effect of suppressed ECT2 expression on cell viability, migratory, and invasive abilities. The results suggested that low expression of ECT2 inhibited the viability (Figure 2(c)) and migratory and invasive abilities of NCI-H2009 cells (Figure 2(d)). Hence, we believed that ECT2 exerted an oncogenic role in LUAD cells.

### 3.3. miR-30a-5p Targets and Regulates ECT2

In order to further explore the molecular regulatory mechanism of ECT2 on LUAD cells, we excavated the upstream regulatory miRNA of ECT2. First, edgeR differential analysis was performed. A total of 186 differentially expressed miRNAs were obtained, including 147 upregulated genes and 39 downregulated genes (Figure 3(a)). The upstream regulatory genes of ECT2 were predicted using the starBase database. The predicted genes were intersected with the previously obtained differentially downregulated miRNAs, and three differentially expressed miRNAs with targeted binding sites on ECT2 were obtained (Figure 3(b)). Pearson's correlation analysis was conducted between ECT2 and these three miRNAs. It was found that miR-30a-5p was negatively correlated with ECT2 and notably downregulated in LUAD tissue (Figures 3(c)–3(e)). High miR-30a-5p expression was associated with the long survival time of patients (Figure 3(f)). In order to make clear the targeted binding relationship between ECT2 and miR-30a-5p, we first used the starBase database to predict the targeted binding sites of ECT2 and miR-30a-5p (Figure 3(g)). Dual-luciferase assay was performed. The results indicated that overexpressing miR-30a-5p could inhibit the luciferase activity of cells with the ECT2 3′-UTR-WT plasmid sequence, but there was no notable change in cells with the ECT2 3′-UTR-MUT sequence (Figure 3(h)), suggesting the targeted binding relationship between miR-30a-5p and ECT2. Subsequently, qRT-PCR and Western blot were conducted to assess miR-30a-5p and ECT2 mRNA and protein levels. The results suggested that the miR-mimic successfully upregulated the miR-30a-5p level and the miR-inhibitor successfully reduced the miR-30a-5p level. When expression of miR-30a-5p was inhibited, the expression of mRNA and protein of ECT2 would increase correspondingly; when miR-30a-5p was overexpressed, the expression of mRNA and protein of ECT2 decreased correspondingly (Figures 3(i) and 3(j)). The above results suggested that ECT2 is the direct target of miR-30a-5p, and miR-30a-5p targets and negatively regulates ECT2.

The article "miR-30a-5p Regulates Viability, Migration, and Invasion of Lung Adenocarcinoma Cells via Targeting ECT2" was retracted in 2023. Reasons: signs of a paper mill; suspected computer-generated content; unreliable results or conclusions; concerns about the data.

### 3.4. miR-30a-5p Inhibits the Viability, Migration, and Invasion of LUAD by Regulating ECT2

A rescue experiment was used to further investigate the effect of the miR-30a-5p/ECT2 axis on LUAD cells. First, the expression levels of mRNA and protein of ECT2 when miR-30a-5p was inhibited alone and when miR-30a-5p and ECT2 were inhibited simultaneously were detected by qRT-PCR and Western blot, respectively. The results indicated that when expression of miR-30a-5p was inhibited alone, the expression levels of mRNA and protein of ECT2 significantly increased; when expression levels of miR-30a-5p and ECT2 were inhibited simultaneously, the mRNA and protein expression levels were notably lower than those of the group inhibiting miR-30a-5p alone (Figure 4(a)). The results of CCK-8 and Transwell assay suggested that compared with the NC group, the viability, migratory, and invasive abilities of NCI-H2009 cells in the group inhibiting miR-30a-5p alone all increased; compared with the group inhibiting miR-30a-5p alone, when miR-30a-5p and ECT2 expression levels were suppressed simultaneously, the viability, migratory, and invasive abilities of NCI-H2009 cells were markedly lower (Figures 4(b) and 4(c)). Therefore, we believe that miR-30a-5p inhibits the viability, migratory, and invasive abilities of NCI-H2009 cells by targeting and regulating ECT2 expression.

## 4. Discussion

ECT2, a protein related to cell viability, is considered to have cancer-promoting effects in lung cancer and other cancers. Xu et al. [12] reported that miR-223 mediated cell proliferation of osteosarcoma cells through the p21 signaling pathway by targeting ECT2. In addition, Hirata et al. [13] revealed that the downregulation of ECT2 expression could effectively suppress the growth of lung cancer cells, and they found that ECT2 also plays a regulatory role in cell cycle progression and cell division. Zhou et al. [14] also found abnormal expression of ECT2 in early LUAD cells, which is considered to be related to the malignant progression of cancer. These findings suggest that ECT2 is highly expressed in LUAD and may play a role in promoting the development of LUAD. In this study, it was revealed by bioinformatics analysis that ECT2 was notably upregulated in LUAD and was markedly correlated with the LUAD clinical stage and pathologic T stage. *In vitro* studies demonstrated that the downregulation of ECT2 expression could significantly suppress the viability, migratory, and invasive abilities of LUAD cells, which was consistent with the trend of previous studies.

In cells, the expression of protein-coding genes such as ECT2 is mostly regulated by noncoding genes, and microRNAs (miRNAs) are one of the crucial regulatory molecules. miRNAs are endogenous small noncoding single-stranded RNAs which are one of the components of the RNA-induced silencing complex (RISC). They recognize the 3′-untranslated region (3′-UTR) of the target mRNA through complementary base pairing and guide the RISC to degrade the target mRNA or suppress the translation of the target mRNA according to the different degree of complementation [15]. Studies manifested that ECT2 is regulated by miRNA in the development of various cancers: miR-194 inhibits cancer cell proliferation by targeting and regulating ECT2 in cholangiocarcinoma [16]; miR-490-5p inhibits metastasis of liver cancer by downregulating E2F transcription factor 2 (E2F2) and ECT2 [17]; miR-223-3p suppresses proliferation, invasion, and migration of breast cancer cells by targeting ECT2 [18]. Therefore, in this study, in order to further explore the specific molecular mechanism of the function of ECT2 in LUAD, we attempted to excavate the upstream regulatory miRNA of ECT2. We screened the bioinformatics data to obtain miR-30a-5p which was abnormally lowly expressed in LUAD tissue and had a targeted binding site on ECT2 mRNA. miR-30a-5p has been manifested to have a tumor-suppressive effect in a variety of cancers. Zhao et al. [19] found that miR-30a-5p is downregulated in prostate cancer and can inhibit cell proliferation by targeting PCLUADF. Quan et al. [20] found that miR-30a-5p inhibits SRY-box transcription factor 4 (SOX4) to inhibit the proliferation, apoptosis, and migration of NSCLC. At present, there are no relevant studies on the effect of miR-30a-5p on the occurrence of cancer by targeting and regulating ECT2. In this study, the targeting relationship between miR-30a-5p and ECT2 was firstly clarified by dual-luciferase reporter assay. Secondly, when the expression of miR-30a-5p and ECT2 was suppressed simultaneously *in vitro*, we found that the promoting effect of inhibiting miR-30a-5p alone on LUAD cell viability was notably restored. Similarly, we found the same situation in the cell migration and invasion experiment; that is, inhibiting the expression of miR-30a-5p and ECT2 simultaneously restored the effect of inhibiting miR-30a-5p alone on the migratory and invasive abilities of LUAD cells. Therefore, we believe that miR-30a-5p can inhibit cell viability, migratory, and invasive abilities of LUAD by targeting and suppressing the expression of ECT2.

The article "miR-30a-5p Regulates Viability, Migration, and Invasion of Lung Adenocarcinoma Cells via Targeting ECT2" was retracted in 2023. Reasons: signs of a paper mill; suspected computer-generated content; unreliable results or conclusions; concerns about the data.

In summary, this study demonstrated that the expression of ECT2 was markedly upregulated in LUAD, while its upstream regulatory miR-30a-5p was downregulated. Moreover, miR-30a-5p can target and suppress ECT2 to inhibit the viability, migration, and invasion of LUAD cells. Therefore, miR-30a-5p and ECT2 may be potential therapeutic targets for LUAD. At the same time, there are also some limitations in this study, such as not verifying the expression of miR-30a-5p and ECT2 in clinical samples and not confirming the effect of miR-30a-5p on the malignant progression of LUAD by the *in vivo* environment. Therefore, further research is still required.

## Figures and Tables

**Figure 1:** ECT2 is upregulated in LUAD. (a) Volcano plot of the differentially expressed mRNAs in the normal group and tumor group from TCGA-LUAD dataset (red dots represent the upregulated genes, while green dots represent the downregulated genes). (b) Differential expression of ECT2 in TCGA-LUAD samples (blue represents normal samples, while red represents tumor samples). (c) Survival analysis of the patients with different expression levels of ECT2 (the blue curve is the low expression group, and the red curve is the high expression group). (d) Box plot of ECT2 expression in different clinical stages of LUAD. (e) Box plot of ECT2 expression in different pathologic T stages of LUAD. (f) qRT-PCR was conducted to detect ECT2 expression in cell lines BEAS-2B, Calu-3, NCI-H2009, and SPC-A1. ∗ represents *p* < 0.05.

**Figure 2:** Downregulating ECT2 inhibits the viability, migration, and invasion of LUAD cells. (a) qRT-PCR was used to detect the expression of ECT2 in each group after transfection (si-ECT2, si-NC). (b) Western blot assay was performed to test protein expression of ECT2 in each group after transfection. (c) CCK-8 assay was performed to detect the viability of cells in each group after transfection. (d) Transwell assay was conducted to detect the migratory and invasive abilities of cells in each group after transfection (×100). ∗ indicates *p* < 0.05.

**Figure 3:** miR-30a-5p targets and regulates ECT2. (a) Volcano plot of the differentially expressed miRNAs in TCGA-LUAD dataset (red dots represent upregulated genes, and green dots represent downregulated genes). (b) Venn diagram of the predicted upstream regulatory genes of ECT2 and differentially downregulated miRNAs in TCGA-LUAD. (c, d) Pearson's correlation analysis between 3 candidate miRNAs (miR-374b-5p, miR-30a-5p, and miR-197-3p) and ECT2. (e) Box plot of the differential expression of miR-30a-5p in TCGA-LUAD samples (blue represents normal samples, while red represents tumor samples). (f) Survival analysis on patients with different miR-30a-5p levels. (g) The binding sites of miR-30a-5p on ECT2 mRNA predicted by starBase. (h) Luciferase activity in different transfection groups detected by dual-luciferase assay. (i) qRT-PCR detected miR-30a-5p and ECT2 mRNA levels in each transfection group. (j) The effects of overexpression or inhibition of miR-30a-5p on protein expression of ECT2 detected by Western blot assay. ∗ represents *p* < 0.05.

**Figure 4:** miR-30a-5p inhibits the viability, migration, and invasion of LUAD by regulating ECT2. (a) The expression of mRNA and protein of ECT2 in each group after transfection (si-NC+NC-inhibitor group, si-NC+miR-inhibitor group, and si-ECT2+miR-inhibitor group) tested by qRT-PCR and Western blot. (b) The viability in each group after transfection detected by CCK-8. (c) The migratory and invasive abilities in each group after transfection detected by Transwell assay (×100). ∗ represents *p* < 0.05.

The article "miR-30a-5p Regulates Viability, Migration, and Invasion of Lung Adenocarcinoma Cells via Targeting ECT2" was retracted in 2023. Reasons: signs of a paper mill; suspected computer-generated content; unreliable results or conclusions; concerns about the data.

**Table 1:** Primer sequences for qRT-PCR.

Primers		Sequences
miR-30a-5p	Forward	5′-ACACTCCAGCTGGGTGTAAACATCCTCGAC-3′
	Reverse	5′-CAGTGCGTGTCGTGGAGT-3′

U6	Forward	5′-CGCGCTTCGGCAGCACATATACT-3′
	Reverse	5′-ACGCTTCACGAATTTGCGTGTC-3′

ECT2	Forward	5′-TCCACTCCAGTTCCTTCA-3′
	Reverse	5′-CGTTGTCCTTCCTCTTCC-3′

*β*-Actin	Forward	5′-GGACTTCGAGCAAGAGATGG-3′
	Reverse	5′-AGCACTGTGTTGGCGTACAG-3′

## Data Availability

The data and materials in the current study are available from the corresponding author on reasonable request.

## References

[1] Siegel R. L., Miller K. D., Jemal A. (2019). Cancer statistics, 2019. *CA: a Cancer Journal for Clinicians*.

[2] Nasim F., Sabath B. F., Eapen G. A. (2019). Lung cancer. *The Medical Clinics of North America*.

[3] Allemani C., Weir H. K., Carreira H. (2015). Global surveillance of cancer survival 1995-2009: analysis of individual data for 25 676 887 patients from 279 population-based registries in 67 countries (CONCORD-2). *Lancet*.

[4] Murata Y., Minami Y., Iwakawa R. (2014). ECT2 amplification and overexpression as a new prognostic biomarker for early- stage lung adenocarcinoma. *Cancer Science*.

[5] Tatsumoto T., Xie X., Blumenthal R., Okamoto I., Miki T. (1999). Human ECT2 is an exchange factor for Rho GTPases, phosphorylated in G2/M phases, and involved in cytokinesis. *The Journal of Cell Biology*.

[6] Yüce O.¨., Piekny A., Glotzer M. (2005). An ECT2-centralspindlin complex regulates the localization and function of RhoA. *The Journal of Cell Biology*.

[7] Wang H. K., Liang J. F., Zheng H. X., Xiao H. (2018). Expression and prognostic significance of ECT2 in invasive breast cancer. *Journal of Clinical Pathology*.

[8] Wang H. B., Yan H. C., Liu Y. (2016). Clinical significance of ECT2 expression in tissue and serum of gastric cancer patients. *Clinical & Translational Oncology*.

[9] Liu B., Yang H., Taher L. (2018). Identification of prognostic biomarkers by combined mRNA and miRNA expression microarray analysis in pancreatic cancer. *Translational Oncology*.

[10] Shi Y. X., Yin J. Y., Shen Y., Zhang W., Zhou H. H., Liu Z. Q. (2017). Genome-scale analysis identifies NEK2, DLGAP5 and ECT2 as promising diagnostic and prognostic biomarkers in human lung cancer. *Scientific Reports*.

[11] Bai X., Yi M., Xia X., Yu S., Zheng X., Wu K. (2018). Progression and prognostic value of ECT2 in non-small-cell lung cancer and its correlation with PCNA. *Cancer Management and Research*.

[12] Xu J., Yao Q., Hou Y. (2013). miR-223/Ect2/p21 signaling regulates osteosarcoma cell cycle progression and proliferation. *Biomedicine & Pharmacotherapy*.

[13] Hirata D., Yamabuki T., Miki D. (2009). Involvement of epithelial cell transforming sequence-2 oncoantigen in lung and esophageal cancer progression. *Clinical Cancer Research*.

The article "miR-30a-5p Regulates Viability, Migration, and Invasion of Lung Adenocarcinoma Cells via Targeting ECT2" was retracted in 2023. Reasons: signs of a paper mill; suspected computer-generated content; unreliable results or conclusions; concerns about the data.

[14] Zhou S., Wang P., Su X. (2017). High ECT2 expression is an independent prognostic factor for poor overall survival and recurrence-free survival in non-small cell lung adenocarcinoma. *PLoS One*.

[15] Bartel D. P. (2009). MicroRNAs: target recognition and regulatory functions. *Cell*.

[16] Gao J., Dai C., Yu X., Yin X. B., Zhou F. (2020). Upregulated microRNA-194 impairs stemness of cholangiocarcinoma cells through the Rho pathway via inhibition of ECT2. *Journal of Cellular Biochemistry*.

[17] Fang Z. Q., Li M. C., Zhang Y. Q., Liu X. G. (2018). miR-490-5p inhibits the metastasis of hepatocellular carcinoma by down- regulating E2F2 and ECT2. *Journal of Cellular Biochemistry*.

[18] Wang X., Tong Z., Liu H. (2019). miR-223-3p targeting epithelial cell transforming sequence 2 oncogene inhibits the activity, apoptosis, invasion and migration of MDA-MB-468 breast cancer cells. *OncoTargets and Therapy*.

[19] Zhao H., Zhang W., Lai X. (2019). miR-30a-5p frequently downregulated in prostate cancer inhibits cell proliferation via targeting PCLAF. *Artificial Cells, Nanomedicine, and Biotechnology*.

[20] Quan X., Li X., Yin Z., Ren Y., Zhou B. (2019). p53/miR-30a-5p/ SOX4 feedback loop mediates cellular proliferation, apoptosis, and migration of non-small-cell lung cancer. *Journal of Cellular Physiology*.

